# Biomechanical Analysis of Different Footwork Foot Movements in Table Tennis

**DOI:** 10.1155/2022/9684535

**Published:** 2022-06-21

**Authors:** Xinrong Li

**Affiliations:** School of Physical Education, Inner Mongolia University, Hohhot 010021, Inner Mongolia, China

## Abstract

In order to solve the problem of athletes with lower limb movement injuries in table tennis footwork, with the increasing risk of sports, the incidence of acute injury also increased. The increase in athletic training, on the one hand, improves the skill level of the athlete; on the other hand, it increases the chances of more chronic injuries. Through the investigation of the injury site of 143 table tennis players, the researchers found that the lower limb injury accounted for 32% of the total injuries and the upper limb injury rate accounted for 33.14% of the trunk, accounting for 34.29%. The injury sites are mostly concentrated in the lumbar region, followed by the shoulders and knees. Through epidemiological research on the injuries of outstanding table tennis players, the survey results show that the probability of lower extremity injuries ranks in the top three, and most of them are acute sprains and chronic strain injuries. By applying the principles of sports biomechanics, a biomechanical analysis of the asynchronous foot movement in table tennis is proposed; from three aspects of kinematics, dynamics, and plantar pressure, it is found that the injury of table tennis is closely related to technical play connect. The risk of sports injury is inevitable in a sense, due to the long-term local overload, which causes the strain of the sports system. In order to avoid or reduce the occurrence of such sports injuries, coaches should standardize the technical movements of the players and arrange the exercise load reasonably according to the characteristics of the sports.

## 1. Introduction

Footwork refers to the movement method of footwork adopted by table tennis players in order to select the appropriate hitting position. Table tennis sports include technique and footwork, both of which are closely related and are indispensable. In training, especially in the early stage of youth enlightenment and basic training, due to the poor mobility of athletes, the main energy of coaches is often focused on cultivating correct techniques, while footwork training is often neglected. The result of this “hands first, footwork later” training results in athletes with good handwork and poor footwork. This affects the progress and improvement of children's sports technology level. Table tennis is a moderate-intensity sport, mainly aerobic metabolism, supplemented by anaerobic metabolism, seen as a healthy form of exercise; it has been accepted by more and more people in leisure and entertainment activities. The three elements of table tennis today are the following: The movement should be fast, the swing power should be strong, and the ball speed should be high. In order to meet the demand for physical fitness in multiround competitive competitions, this requires athletes to increase exercise load and improve motor units in their usual training. Moreover, in the physical training, the focus is on the strategic idea of “focusing on special physical training,” effectively giving play to the physical fitness of athletes and making reasonable use of special endurance to improve competition performance. Scholars have found that, in the multiball practice of table tennis, the dynamic balance ability of the body will decline with the extension of training time, which will affect the performance level of players, and, compared with male table tennis players, female players will have an earlier decline in balance ability. Regarding the study of table tennis footwork, relevant scholars from various countries have actively integrated the advantages of various disciplines to analyze their in-depth mechanism. Athletes of different skill levels were selected to carry out systematic comparative research to reveal the internal laws and external connections of footwork itself. Using the improved letter notation method, the touchdown sequence of various footwork was analyzed from the perspective of footwork sequence, and the relationship between footwork, technique, and landing point was found. Sports biomechanics has become a powerful method for research in this field, modeling foot skeletal muscles based on software such as V3D, CAD, and finite element, and researchers can use a variety of measurement methods to obtain more detailed data on the foot and use computers for processing and analysis. The author aims to apply the principles of exercise biomechanics, from the three aspects of kinematics, dynamics, and plantar pressure, in addition to an in-depth study of the three footsteps in table tennis: the biomechanical laws of foot movement in stride, parallel step, and cross step; the following main conclusions are drawn: Forehand stride and forehand side-by-side strike have similar movement forms of the foot after the force foot hits the ground. There are similarities in the movement of the foot after the backhand step; the backhand side step and the backhand cross step hit the ball with the force foot on the ground. Among the three footwork movements, the movement form of the foot is similar when the pedal is extended off the ground when hitting the ball. Among the three footwork movements, the peak force of the vertical reaction force on the ground and the load rate of the force when the athlete completes the cross step are the largest; moreover, the flexion and extension range of the stepping joint of the force-generating foot and the change range of the heel angle are the largest; therefore, the frequent use of cross gait by athletes may increase the risk of foot fatigue injury. In the three kinds of footwork movements, when the peak force of the vertical reaction force of the ground on the hitting foot appears, the foot is in the flipping motion before and after the maximum valgus angle occurs; coupled with the maximum dorsiflexion state of stepping on the joint at this time, the probability of joint movement injury is increased. During the typical footwork of table tennis, the main bearing area of the plantar pressure of both feet is concentrated in the forefoot area, and the force in the midfoot area is not obvious. The peak value of plantar pressure in the rear area of the foot when hitting the ball was the largest, followed by the parallel gait, and the stride gait was the smallest. The middle area of the forefoot is a relatively stable main force area of the forefoot area, and the magnitude of the peak plantar pressure on the lateral area of the forefoot and the medial area of the forefoot is related to the action form of the gait, as shown in Figure 1.

## 2. Literature Review

Since the beginning of the 21st century, Cf, A. et al. said that, with the fusion of various play styles, the sport of table tennis continues to develop in a fast and ferocious direction, requiring players to have outstanding expertise and comprehensive technology, be proactive, and be the first to get started [1]. In particular, the ITTF proposed three new rules in 2000: The sphere is changed from 38 mm to 40 mm; the 21-point system is changed to an 11-point system; the two-point rotation method and unobstructed serving are implemented in the serving rules. These rules place higher demands on table tennis players in various aspects. Shao et al. feel that as the competition becomes more and more confrontational and the ball turns more and more, the technical requirements for the movement range and direction of the athlete are also more refined, so that the athlete's footwork has become the decisive factor in the game [2]. Former Japanese world champion Nobuhiko Hasegawa had a famous quote: “Footwork is the life of table tennis.” It can be seen that table tennis footwork plays a vital role in the completion of the entire hitting action and the rationality, as well as effectiveness and scientificity of the completion of the action. Ardiyanto et al. felt that, in the study of table tennis footwork, the methods and theories of biomechanics provided a scientific means and basis for it [3]. The research scope of biomechanics includes the whole human body, and the research of foot biomechanics is an important part of it. The rise of foot biomechanical research is the result of several factors. Davide et al. said that, first, from a clinical point of view, with the continuous improvement of diabetes treatment methods, it has become possible to prolong the life of patients as much as possible, but, at the same time, the incidence of diabetic complications of diabetic foot is also increasing, medical workers are eager to know the causes of pathological phenomena such as diabetic foot, and biomechanics has begun to enter this field of research [4]. Second, in the work of Hong and Chao, from the perspective of the market, with the rapid development of competitive sports, the scientific scope of competitive sports has become more and more extensive, and the impact of sports shoes on sports has also received increasing attention; people have higher and higher requirements for the injury prevention ability and functional performance of special sports shoes, and it is particularly important to study the biomechanical characteristics of the foot in different special sports [5]. Finally, from a technical point of view, electronic measurement technology and computer technology provide a possibility for the study of foot biomechanics. Researchers can use a variety of measurement techniques to obtain plantar pressure and ground reaction force, process them with computers, and use CAD systems and professional finite element analysis software to model and analyze the foot. Bańkosz and Stefaniak said that “footwork is the soul of table tennis” and accurately summarized the importance of footwork movement in table tennis [6]. Footwork is an important part of table tennis batting and the beginning of each action, and the source of strength comes from the feet and legs. Wu et al. felt that when table tennis players take the initiative to attack the ball, in order to improve the quality of the shot, the movement of the upper limbs alone is not enough [7]. In other words, superb ball skills depend on precise footwork movement, and agile hitting awareness is achieved by flexible, fast, and stable footwork. Sports biomechanics is a common method used in table tennis footwork research; Li et al. felt that, using the theory of exercise biomechanics, in order to explore the biomechanical differences of the dominant foot between professional athletes and beginners in table tennis parallel gait and cross gait, the results and conclusions can improve the in-depth understanding of table tennis footwork for coaches and athletes and then promote the scientific development of table tennis footwork. Previous studies have mainly focused on the three-dimensional motion of human large joints, while the biomechanical characteristics of small foot joints in table tennis footwork have not yet been revealed [8]. Until the Oxford Foot Model (OFM) was discovered, the skeletal muscle model of the small joints of the foot was widely used. Tang et al. said that the Oxford Foot Model is improved on the basis of the traditional Plug-in-Gait model. This model provides more details of the foot and is a reliable multistage study of foot movement [9]. The research of this model mostly focuses on the motion analysis of the forefoot, hindfoot, and great toe, the three-dimensional motion of the forefoot relative to the hindfoot, and the hindfoot relative to the tibia, and the motion of the big toe on the sagittal plane is more detailed. In the analysis of a large number of movement patterns, the model can be widely used in foot analysis in sports and clinical medicine. Therefore, Tabrizi et al. think that using the Oxford Foot Model to study the foot biomechanical characteristics of table tennis footwork can find more movement patterns between the small joints of the foot and help us deeply understand its movement mechanism, which will be a brand new attempt [10].

## 3. Research Method

Based on the modeling and analysis of human kinematics, the author proposes a new marker point setting scheme and a gait motion measurement system composition scheme; research will be conducted on key techniques for gait motion measurement using established protocols, that is, to study how to obtain lower limb geometric parameters and gait kinematic parameters from gait measurement data. In the traditional gait motion measurement method, the position of the joint center (or axis) is calculated according to the coordinate position of a series of anatomical key points, combined with the manually measured geometric dimensions of the lower limbs. The positions of these anatomical key points are represented by physical measurement identification points on the skin surface or designated points (or virtual identification points) in the calibration process. Therefore, the accuracy of anatomical key point positioning in traditional measurement methods will directly affect the identification of joint positions; as a result, the accuracy and repeatability of gait motion measurement are affected, and the manual positioning process of anatomical key points is also a key factor affecting the pretest preparation time. Firstly, the fitting algorithm of joint position and model geometric parameters is established by analyzing the motion constraint relationship of lower limbs; then, the extraction algorithm of gait motion parameters is established by sampling inverse kinematics analysis method. For the implementation of this algorithm, algorithms and technical support are provided for marker point setting schemes and measurement methods, so that gait measurement does not depend on manual positioning of anatomical key points. Finally, through experiments and analysis of the experimental results, the feasibility of the gait measurement system and related algorithms proposed by the author is discussed [11]. When processing and analyzing the sampled data, it is often necessary to calculate the average posture of the lower limb movements, for example, attitude calculation of measuring rigid body under standard standing posture and attitude filtering. In the space three-dimensional coordinate system, the attitude description of the rigid body can take many forms, such as the direction cosine matrix, the finite rotation quaternion coordinate, the Euler quaternion coordinate, the Euler angle coordinate, and the Cardan angle coordinate. The general algorithm for the weighted average of vectors or matrices is shown in the following formula [12, 13]:

(1) $$\begin{array}{c} A=\frac{\sum_{i=1}^{n}w_{i}A_{i}}{\sum_{i=1}^{n}w_{i}}. \end{array}$$

The Lifemod interface software of Python language is used to convert Motion's 6 pieces of data and 2 pieces of kinematics data obtained from analysis and generate Slf files that Lifemod can recognize. The height, weight, and other information of the subjects were input, and the 19-link human model was established through Lifemod's own human morphology database. The posture adjustment after data is given. The collected kinematic data is given to the model, and then, through posture adjustment and balance analysis, the floor pad model is established, and the contact between the human body model and the floor pad is established. The contact force between the human body model and the floor pad model, the force and moment of each link of the human body model, and the kinematic index of each link were simulated for 1 s to obtain 1000 pieces of data, which was the same as the acquisition frequency of the force table [14]. Formula (1) of inertia for strength training is shown below:

(2) $$\begin{array}{c} j\theta +k\theta =T\left(t\right), \end{array}$$

where *A* is the weighted average matrix of matrix *Ai* (*i* = 1, 2, ..., *n*) and *Wi* is the weight of *Ai*. However, if the mean value calculation of the direction cosine matrix also adopts the above method, then the resulting matrix will no longer satisfy the constraints of the directional cosine matrix. Euler quaternion coordinates, Euler angle coordinates, and Cardan angle coordinates cannot use a simple weighted average to calculate the average attitude; this is mainly because these pose coordinates are essentially rotation vectors rather than ordinary vectors. Among the attitude coordinates, Euler quaternion is widely used because of its small calculation amount, nonsingularity, and full attitude work. Wahba proposed constructing the cost function to solve the Euler quaternion mean value problem in the 1960s; based on this idea, many researchers have proposed various algorithms. Among them, Markley et al. directly used the direction cosine matrix as the object to solve the weighted mean quaternion method, because the singular value decomposition of the matrix is not involved, making the algorithm relatively simple and widely used. The Euler quaternion *n* is a four-dimensional vector as shown in the following formula:

(3) $$\begin{array}{c} \underline{\Lambda }={\left(\lambda_{\text{0}},{\underline{\lambda }}^{T}\right)}^{T}={\left(\lambda_{\text{0}},\lambda_{1},\lambda 2\text{,}\lambda_{3}\right)}^{T}, \end{array}$$

where *λ* is the vector part and *λ*_0_ is the scalar part. Since the Euler quaternion is essentially a rotation vector and its four variables are not independent, it must satisfy the normalization constraint as shown in the following formula:

(4) $$\begin{array}{c} \underline{\Lambda^{T}}\underline{\Lambda }={\left\|\underline{\Lambda }\right\|}^{2}=\lambda_{0}^{2}+\lambda_{1}^{2}+\lambda_{2}^{2}+\lambda_{3}^{2}=1. \end{array}$$

The direction cosine matrix corresponding to the Euler quaternion $\underline{\Lambda }$ is shown in the following formula:

(5) $$\begin{array}{c} \underline{A}\left(\underline{\Lambda }\right)=\left(2\lambda_{0}^{2}-1\right){\underline{I}}_{3}+\underline{\lambda }{\underline{\lambda }}^{T}+2\lambda_{0}\overset{∼}{\underset{-}{\lambda }}, \end{array}$$

In order to calculate the average Euler quaternion, construct the pose matrix cost function as shown in the following formula:

(6) $$\begin{array}{c} \bar{\underline{\Lambda }}=\arg\min\sum_{i}w_{i}{\left\|\underline{A}\left({\underline{\Lambda }}_{i}\right)\right\|}_{F}^{2}. \end{array}$$

From the definition of the Frobenius norm and the orthogonality of the directional cosine matrix, the following formula can be obtained:

(7) $$\begin{array}{c} {\left\|\underline{A}\left(\underline{\Lambda }\right)-\underline{A}\left({\underline{\Lambda }}_{i}\right)\right\|}_{F}^{2}=6-2tr\left[\underline{A}\left({\underline{\Lambda }}_{i}\right)\right]. \end{array}$$

The time series of foot position coordinates and posture coordinates is the motion curve of the foot, and the position coordinates can be represented by the position coordinates of the stepping joints; the posture coordinates are represented by the direction cosine matrix of the foot conjoined base *e*4 with respect to the reference base or other posture coordinates. Corresponding to each sampling point, the changes in the position and posture of the foot in the pelvic conjoined base *e*1 are calculated; the following focuses on the motion curve of the foot in the overall base. For any sampling point, the direction cosine matrix *A*04 of the foot conjoined base *e*4 with respect to the overall base *e*0 is obtained. The position vector of the stepping joint in the overall base dream can be expressed as in the following formula:

(8) $$\begin{array}{c} r_{\text{ankle}}=r_{4b}-d_{\;}. \end{array}$$

Due to the influence of the model error, the actual lower limb joints are not truly pivoted, making it difficult to obtain accurate and consistent results for the fitting of the position of the joint rotation center (or rotation axis). For example, the movement pattern of the knee joint is not a simple flexion and extension movement; rather, it is a complex multi-DOF mode that combines flexion, roll, slide, lateral shift, and axial rotation. The flexion and extension movements do not revolve around the same center of rotation but generate multiple instantaneous centers of rotation according to the movement process. During the process of extending and flexing the knee joint, if the instantaneous center of rotation of each movement is continuously marked, the form one on the femoral bone, +*J*”-shaped trajectory, taking the lateral femoral skeleton as a reference, analyzing the electronic *X*-ray films at 9 different positions of the knee joint of 5 volunteers, and measuring the straight-line distance from the joint measurement axis to the lateral skeleton at each position, the measurement results are as follows: With flexion 40” as the center, the distance from the joint measurement axis to the lateral femoral skeleton gradually increases; the greater the flexion angle, the farther away from the lateral femoral skeleton, and the joint measurement axis in the entire range of motion is the same as that on the outer skeleton. The intraclass correlation coefficient (ICC) is often used to evaluate the reliability of a single measurement parameter, but it is not suitable for the repeatability evaluation of the entire curve or waveform; the evaluation index of the repeatability of the gait motion curve is called the adjusted coefficient of multiple correlation (CMC) or the adjusted coefficient of multiple determination (CMD). This method has been used by many researchers in related research. The CMC method is used to analyze the repetition reliability of joint motion parameters as shown in the following formula:

(9) $$\begin{array}{c} R_{wt}^{2}=1-\frac{\sum_{i=1}^{M}\sum_{j=1}^{N}\sum_{t=1}^{T}{\left(Y_{ijt}-{\bar{Y}}_{it}\right)}^{2}/MT\left(N-1\right)}{\sum_{i=1}^{M}\sum_{j=1}^{N}\sum_{t=1}^{T}{\left(Y_{ijt}-{\bar{Y}}_{i}\right)}^{2}/MT\left(N-1\right)}. \end{array}$$

The value of the curve is obtained by the *J*th test (trial) in the *i*th experiment in *Y*_*ijt*_ at the sampling point *t*; *T* is the total number of adopted points contained in the curve; *N* is the total number of trials for each subject in each experiment; in this experiment, *N* = 3; *M* is the total number of experiments (tests) for each subject, and *M* = 4 in this experiment; *Y*_*it*_ and *Y*_*i*_ are shown in the two following formulas:

(10) $$\begin{array}{c} Y_{it}=\frac{1}{N}\overset{N}{\underset{j=1}{\sum }}Y_{ijt}, \end{array}$$

(11) $$\begin{array}{c} Y_{i}=\frac{1}{NT}\overset{N}{\underset{j=1}{\sum }}\overset{T}{\underset{t=1}{\sum }}Y_{ijt}. \end{array}$$

The algorithm studied by the author is the key technology of the gait measurement system, which overcomes the limitations of the traditional gait measurement system. The realization of this technology makes the marking point layout of the gait measurement system independent of the manual positioning of anatomical key points, and the length of the lower limbs does not need manual measurement, so that the measurement method with fewer marking points can be realized, thus simplifying the measurement process, and, at the same time, it is helpful to reduce the influence of human error caused by the arrangement of marker points and improve the reliability of repeated measurement between experiments.

## 4. Experiments and Analysis

The stride method includes a forehand step and a backhand step. The experimental subjects all shoot with the right hand, move the right foot to the right for a forehand stride, and move the left foot to the left to perform a stride action during a backhand stride. Among them, the stride foot is the main moving foot that constitutes the stride gait, and it is also the main force-generating foot to complete the batting action, and, according to the research needs, the left foot (i.e., the supporting foot) in the forehand step is called the moving auxiliary foot, and the right foot (i.e., the stepping foot) is called the hitting force foot. The right foot in the backhand step is called the moving auxiliary foot, and the left foot is called the hitting force foot.  Figure 2 shows the average-time curve of the flexion and extension angle, heel key angle, and toe extension angle during the forehand stride action of all subjects. As can be seen from Figure 2, when the subjects performed the forehand stride action, when the ball hit the ground, the foot basically did not turnover. However, after landing, the center of gravity of the body shifts to the foot where the ball is used, and the force on the foot increases and turns into a valgus state; when the calcaneal angle decreases and reaches the minimum value, that is, the maximum valgus angle, the stomping, flexion, and extension angle increases, and the restless joint performs hesitant movement. After the heel angle reaches the maximum valgus angle, it begins to increase; when the first peak force occurs, the foot is doing varus movement, the stomping joint is in the dorsiflexion movement, the toe extension angle decreases rapidly, and the foot that hits the ball with force enters the center of gravity adjustment stage of full-foot support.

The first stress stage is over, and the batting force foot enters the second stress stage. With the active push and extension of the hitting force foot, the force on the foot increases, the Achilles tendon angle begins to decrease, the foot performs valgus movement, and the restless joint continues to do dorsiflexion movement; when the foot reaches the maximum eversion of the second force stage and the manic joint reaches the maximum dorsiflexion angle, the second peak force appears. After hitting the ball, the force foot starts to push and extend off the ground, the stomping flexion and extension angle increases, and the restless joints do active flexion movement, and the maximum flexion angle is reached at the moment of lifting off the ground. In the stage of kicking off the ground, the toes and the toe joints land on the ground, and the heel is lifted; the toes begin to make the maximum toe extension movement around the toe extension joint, the calcaneal angle increases with the increase of the extension angle of the toe, and the foot performs a varus motion, which changes from the everted state to the initial state at the time of landing [15]. In the kinematic analysis of backhand stride action, all subjects performed backhand stride action when subjects performed backhand stride action, the force on the foot increased after hitting the ball with the force of the foot on the ground, and the foot turns into a valgus state and reaches the maximum valgus angle; at the same time, the stomping flexion and extension angle decreases. The manic joints do dorsiflexion movement; in the landing stage, the heel and toe joints land on the ground, and when the toes are off the ground, the toes begin to make the maximal toe extension movement around the toe joint; the toe extension angle increases first and then decreases before the toe hits the ground. When the first peak force appeared, the foot was in varus state and continued to do varus motion, and the pedal joint reached the maximum dorsiflexion angle. At this time, the extension angle of the toe decreases, and the hitting force foot enters the adjustment stage of the center of gravity supported by the full sole of the foot. Step on the joint to adjust the extension and flexion of a small angle, begin to do the valgus movement, and the toe extension angle enters the plateau phase of change. After the hitting force foot enters the second force stage, the force on the foot increases, the foot continues to do valgus movement, and the restless joint is adjusted in the form of dorsiflexion; when the second peak force occurs, the pedal joint reaches the maximum dorsiflexion angle of the second force stage, and the foot is in a valgus movement. After hitting the ball, the force foot starts to push and extend off the ground, the stomping flexion and extension angle increases, and the restless joints do active flexion and flexion, and the maximum kick angle at the moment of leaving the ground is reached. The toes begin to make the maximum toe extension movement around the toe joint, the extension angle of the toe increases, and the foot performs varus movement at the same time, from the eversion state to the initial varus state at the time of landing. It can be seen from the analysis of the plantar pressure of the stride gait that the main bearing area of the plantar pressure of both feet in the support stage is the forefoot area, and the pressure peak in the forefoot area is. The percentage reaches around 50% [16]. The stress on the midfoot area is not significant, the peak pressure is only about 30% of the body weight, and the peak pressure only accounts for about 15–18% of the total of the three areas. The peak pressure on the back of the foot during the support phase exceeds half of the body weight, but it is not as pronounced as that on the front of the foot. The step-step method is mostly used in the fast-break game near the table, counterattacking the ball from a large angle in the forehand position; when the subject moves to the forehand position with the forehand stride, in order to meet the near billiards, the body's center of gravity moves toward the near table; at this time, the force on the forefoot area is increased relative to the rear area, so the force on the forefoot area is the most obvious relative to each area during the forehand step; the same is true for the force on the sole of the backhand stride [17]. Comparing the mobile auxiliary foot with the batting force foot, there was no significant difference in the force in the midfoot area between the two, and the force in the forefoot area was greater when hitting the ball; the force of the auxiliary foot in the rear area of the foot is greater than that of the ball-hitting force [18, 19]. Because the batting force foot also undertakes the task of actively pushing and extending the force to participate in the batting action and returning to the original position, at this time, the forefoot area, which is the main force-bearing area of the kicking and stretching action, bears more pressure. However, the mobile auxiliary foot is in a state of full-foot support most of the time during the entire forehand step, and the force is relatively scattered; therefore, the difference between the force of the forefoot area and the rear area of the mobile auxiliary foot is small. Through the comparative analysis of the support time of the subjects' hitting power foot, it is found that the stride footwork action has more support time than the parallel footwork; this is because the movement speed and rhythm of the parallel footwork are faster than those of the stride footwork, and the ball-strengthening foot transitions to the active kick off the ground faster in the support phase. After the cross footwork action hits the ball with the force foot on the ground, wait until the mobile auxiliary foot moves the landing support and adjusts the body posture to the direction facing the initial position and then starts to actively push off the ground; therefore, the cross gait method is more complicated, and the support time of the hitting force foot is significantly longer than those of the stride gait method and the parallel gait method, and the difference is significant as shown in Figure 3.

As can be seen, the maximum load rate of the vertical reaction force on the ground after the strike force foot hits the ground in the cross-gait action is significantly larger than those of the stride gait and the parallel gait, and the difference is significant. This is because the first peak force after hitting the ball in the cross footwork is the largest among the three footwork movements, and its appearance time is also the earliest; the hitting force foot should reach the maximum first peak force in the shortest time as shown in Figure 4.

It can be seen that, among the three steps, after the cross footwork hits the ball with the power foot on the ground, the first peak force of the vertical reaction force from the ground is significantly larger than those of the other two footwork types. Due to the cross footwork, the batting force foot is in the single support stage for a period of time after landing, and the body weight is concentrated on the batting force foot, coupled with a large range of rapid movement, resulting in a high landing influenced by factors such as speed; as a result, in the action of the cross footwork, the first peak force of the hitting force foot in the first force stage is significantly greater than those of the other two footwork types. In the process of kicking off the ground after completing the hitting action, the distance back to the initial position of the cross footwork action is farther than those of the other two footwork types; compared with the other two types of footwork, the time left for the adjustment of the cross footwork between the two strokes is less, and the second peak force experienced is the largest [20], as shown in Figure 5.

The change range of the foot angle reflects the movement range of the subject's hitting force during the support force stage; with greater movement range of each link of the foot, especially in the state of continuous force, the risk of sports injuries increases accordingly. Athletes have the greatest flexion and extension of the restless joints during the cross-step process. The previous research on the change law of the angle of flexion and extension in the support stage of the hitting force has shown the maximum changes in the flexion and extension angles of the three footwork movements; they all appeared in the final stage of kicking and extending off the ground, reflecting the significant role of the kicking and flexing movement of stepping on the joint in the process of kicking and extending off the ground. In the action of cross footwork, the kicking foot is in the stage of kicking and extending off the ground, it is necessary to overcome greater resistance than the other two footsteps to return to a farther initial position, and the flexion movement of stepping on the joint is more important, and the range of motion is greater [21]. Therefore, the change range Δ*α* of the angle of flexion and extension in the support stage of the impacting foot in the cross-footwork action is larger than those of the other two footwork types, and the difference is significant. There was no significant difference in the change range Δ*γ* of the toe extension angle of the hitting foot when the subjects performed the three footwork movements, and the uniformity of the three footwork movements is not large, indicating that the toe extension movement of the hitting force foot in the process of supporting the force is not affected by the asynchronous movement, and the toe extension angle only changed within a small angle range, and there was no obvious movement of the toe extension. The heel angle is an important index to reflect the flipping of the foot during exercise, and the magnitude of its variation Δ*β* is also an important reference index to evaluate the probability of sports injuries. As can be seen from Figure 6, the change amplitude Δ*β* of heel angle in the cross-gait action is significantly larger than those of the step-step and parallel gait, and the difference is significant. This may be because the cross footwork strikes the force foot away from the incoming ball, and the relative position of the strike force foot at the time of landing is beyond the body in the incoming ball direction, coupled with factors such as the faster initial speed before landing after a long moving distance; the results are shown in Figure 6.

From the previous results, it can be found that when the subjects perform the three footwork movements, there is a large change in the key angle in the support stage of the hitting force foot; most occur in the valgus movement of the first stress stage and the varus movement of the second stress stage. Comparing the kinetic data, it can be found that the maximum valgus angle of the heel angle mostly occurs near the time when the first peak force occurs in the first stress stage, which means that the foot is subjected to a large vertical force when the foot is in the valgus state, and the impact of the reaction force will increase the probability of foot sports injury [22, 23]. The maximum varus angle of the heel angle mostly occurs at the moment of kicking off the ground, with the appearance of the maximum extension angle of the restless joint; at this time, the hitting force foot is about to leave the ground, and the force is very small. As can be seen, the maximum varus/valgus angles of the power foot in the cross-footing action were larger than those in the other two footwork types, and the difference was significant. The results of the previous study also showed that, during the process of the subjects' performing, the three footwork movements and the peak force of the hitting force foot in the support stage occur during the maximum dorsiflexion angle of the manic joint and the rapid turnover of the foot. In order to prevent sprains from stepping on joints, limit the force acting on the anterior ligament of the talus during stomping, the design of the shoe must strive to limit the varus and valgus forces acting on the restless joint, and this external twisting force is maximized during flexion. In addition, since the stomp joint has a certain degree of lateral flexibility when the stomp joint is flexed, this reduces its own stability; therefore, in order to provide support for sports shoes to resist the varus force that frequently causes sprains, sports shoes must provide stability to counteract the rotation of the pedal joints, especially in the flexion state. Based on the experimental results, the smaller joint range of motion of professional table tennis players when they complete the parallel footwork proves that professional athletes have better foot control and technical stereotypes [24]. For professional athletes, a larger internal rotation of the rear foot at the end of the lead can help the players to complete the gait better, and, with the larger abduction of the forefoot, it is beneficial to maintain the stability of the body's center of gravity. In addition, using V3D technology and high-speed cameras, we found that, during Phase I footwork movement, professional table tennis players are used to landing on the rear foot area, while beginners use the front corner area. This also explains why, during this process, the peak pressure of professional athletes occurs in three areas of the medial and lateral hindfoot and the lateral forefoot; for beginners, peak pressure occurs in three different areas: the big toe, the medial forefoot, and the middle. At the same time, this finding can illustrate that professional athletes can better distribute the body's center of gravity on the entire sole plane, providing a more stable swing foundation for the next stage [25, 26]. At the end of the lead-in period, professional athletes showed less hindfoot varus and forefoot valgus and greater extension of the big toe, which was beneficial to better maintain the balance of the center of gravity and adjust the posture for the rapid transition to be prepared to the next stage. From the results of the study, it was found that professional athletes have a more stable body weight transfer ability in the parallel gait. Professional athletes showed significantly greater dorsiflexion in the forefoot, relative to the hindfoot and relative to the tibial angle of the hindfoot than beginners. According to the systolic relaxation theory, the elastic potential energy previously stored in tendon extension can increase the concentric contraction of the muscle, which means that the professional table tennis player's greater dorsiflexion during the full lead phase can store more energy for the swing phase. The limitations of the author's study are manifested in the following aspects: First, the author's study lacked a gender-specific comparison of parallel gait and cross gait due to limitations in recruiting subjects [27]. Another potential limitation is that there are large differences in training years, although all professional table tennis players have the same level of skill level and are from the same university table tennis team, but this may limit the validity of the experiment to some extent [28]. In addition, beginners have different degrees of differences in their learning ability; this may affect the effectiveness of gait learning. Second, only the differences in the biomechanics of the dominant leg were compared. In fact, the nondominant leg also plays an important role in maintaining body stability during the swing phase. Finally, this experiment is to simulate the footwork movement process in actual combat, not in real competitive competitions. Considering a series of uncontrollable factors (athlete psychology, unfixed table tennis balls, etc.) will affect the results of the experiment.

## 5. Conclusion

Research shows the following: Compared to beginners, professional athletes spend less time performing side-step and cross-step footwork and show a smaller range of motion and faster angular velocity. This verifies that professional athletes have better ability to use foot drive and body balance in footwork movement techniques. At the end of the lead-up period, professional athletes in the gait show less forefoot valgus and hindfoot varus and greater flexion of the big toe, and the cross gait shows a smaller forefoot flexion and abduction angle, which is conducive to maintaining the stability of the body's center of gravity. For professional athletes, larger peak pressures and relative loads were found in the lateral forefoot and medial-lateral hindfoot regions in these two table tennis footwork styles. The results and analysis of this study are beneficial to provide more valuable theoretical reference for coaches and beginners in the process of footwork training and in the use of parallel and cross gait, how to use foot movement to improve the quality of technical movements and how to maintain body stability, and there are lessons to be learned. The author reveals in detail the kinematics and dynamics of the foot in the three footwork movements of table tennis, which provides data and theoretical basis for improving the effect of footwork movements and preventing foot injury in table tennis players. The movement forms of the foot after the forehand stride and the forehand parallel strike are similar. There are similarities in the movement of the foot after the backhand step, the backhand side step, and the backhand cross step hit the ball. In the three footwork movements, the motion forms of the feet when the pedals are extended and lifted off the ground are similar. The cross footwork is the longest, the stride footwork is the second, and the footwork is the shortest. In the cross-footwork method, the ball-strengthening foot is in the middle of the support stage, and the body posture and the center of gravity adjustment stage appear to be obviously unstressed or less stressed. Among the three footwork movements, the peak force of the vertical reaction force on the ground and the load rate of the force when the athlete completes the cross step are the largest; moreover, the flexion and extension range and calcaneal angle of the force-generating foot have the largest changes; therefore, the frequent use of cross gait by athletes may increase the probability of foot fatigue injury. In the three kinds of footwork movements, when the peak force of the vertical reaction force of the ground on the hitting foot appears, the foot is in a flipping motion before and after the maximum valgus angle occurs, coupled with the maximum dorsiflexion state of the stepping joint at this time, and the probability of injury of the stepping joint is increased. The main bearing area of the plantar pressure of the feet in the three gait movements is concentrated in the forefoot area, and the force in the midfoot area is not obvious. The peak value of plantar pressure in the rear area of the foot when hitting the ball was the largest, followed by the parallel gait, and the stride gait was the smallest. The middle area of the forefoot is the relatively stable main force area of the forefoot area, the peak size of the plantar pressure on the lateral area of the forefoot and the medial area of the forefoot is related to the action form of the footwork, the main force-bearing area of the forefoot area. The peak force of the ground reaction force received by the power foot in the buffering stage and the kicking stage of the three footwork movements is relatively large; therefore, special sports shoes for table tennis should have appropriate shock absorption and buffering functions, in order to relieve the load of frequent impact force on the feet of table tennis players during the game. The peak force of the three footwork movements hitting the power foot in the support stage appears in the maximum dorsiflexion angle of the restless joint and the rapid turnover of the foot. Therefore, special sports shoes for table tennis need to provide good stability support for the stepping joint to resist the foot in the support stage, especially in the state of stepping and bending, and the frequent torsional external force will reduce the probability of foot sports injury. Table tennis footwork action is the active and rapid exertion of the power foot in the stage of kicking off the ground; special sports shoes for table tennis are required to have good energy return performance, providing better conditions for table tennis players to move quickly.

## Figures and Tables

**Figure 1:** Biomechanical analysis of asynchronous foot movement in table tennis. The middle area of the forefoot is a relatively stable main force area of the forefoot area, and the magnitude of the peak plantar pressure on the lateral area of the forefoot and the medial area of the forefoot is related to the action form of the gait.

**Figure 2:** The average-time curve of each angle of the forehand stride strike. The right foot in the backhand step is called the moving auxiliary foot, and the left foot is called the hitting force foot.

**Figure 3:** Comparison of the average support time at Farley corners. After the cross-footwork action hits the ball with the force foot on the ground.

**Figure 4:** Comparison of the average value of the maximum load rate of the vertical reaction force on the ground of the hitting force. The difference is significant.

**Figure 5:** Comparison of the average value of the first peak force and the average value of the second peak force of the mana foot for three footwork strokes. Comparison with the other two types of footwork.

**Figure 6:** Comparison of the average value of the variation amplitude of the foot angles of the three gait styles, coupled with factors such as the faster initial speed before landing after a long moving distance.

## Data Availability

The data used to support the findings of this study are available from the author upon request.
